The article "Network Fault Diagnosis of Embedded System Based on Topology Constraint and Data Mining" was published in 2022. Journal: Comput Intell Neurosci.

# Network Fault Diagnosis of Embedded System Based on Topology Constraint and Data Mining

**DOI:** 10.1155/2022/1868677

**Published:** 2022-02-17

**Authors:** Tao Zhang

**Affiliations:** School of 3D Printing, Xinxiang University, Xinxiang 453000, Henan, China

## Abstract

Maintaining the safe and efficient operation of network technology is an important development task of the computer industry. Topology constraint can optimize and combine the tracking results and select the target objects with better tracking performance to obtain the final tracking results and determine the target scale changes. Data mining technology can reduce the number of combinations to be detected, reduce the workload, and improve the timeliness and accuracy of the process of mining alarm association rules. Therefore, based on the summary and analysis of previous research results, this paper studied the network fault diagnosis of the embedded system method based on topology constraint and data mining. Firstly, a fault diagnosis topology model was established by constructing a topology search algorithm, which eliminated the filtering of association rules without topology relationship; the association rule-based data mining model was analyzed through the collection of network alarm data; the model algorithm was applied to the simulation experiment of network fault diagnosis of the embedded system and achieved good results. The results show that correcting rage of retrieval varies from 0.65 to 090 under different window sizes; the running time of the proposed method drops from 310 s to 35 s during 1–8 step/s of the sliding step, while the node degree ranges from 8 to 14 and diagnostic accuracy ranges from 0.97 to 0.94; the remaining alarm number increases from 0.5 to 3.5 threshold value, while the regular association number distributed in an interval of 40 to 140. The algorithm in this paper provides a reference for further research on network fault diagnosis of the embedded system.

## 1. Introduction

With the rapid development of network information, the structure of computer networks is becoming more and more complex, the application fields are becoming more and more extensive, and people are increasingly dependent on the network. Therefore, the security and reliability of the network have become more and more important. As the main way to obtain the fault of the modern computer network and diagnose the system fault, the log uses the log information generated during the network operation to diagnose the fault, which has become a research hotspot of network fault diagnosis of the embedded system. Because there is a nonlinear mapping relationship between the fault type and the fault feature, the fault information has uncertainty. As the network architecture scale increases, a large amount of log information is generated during the running process, and the fault feature extraction is very useful, thus increasing the difficulty of fault diagnosis [1]. In the existing fault diagnosis methods, the artificial neural network-based method has good fault tolerance, and it is not necessary for the domain experts to summarize the empirical rules of the diagnosed system from the domain knowledge or case, which is beneficial to overcome the knowledge based on the symbolic reasoning method. Obtaining bottlenecks, unlike symbol-based reasoning methods, which are sensitive to errors in rules or models, supports parallel computing. As parallel technology and hardware developments have become more widely used, they have been used to implement fault diagnosis [2].

The article "Network Fault Diagnosis of Embedded System Based on Topology Constraint and Data Mining" was published in 2022. Journal: Comput Intell Neurosci.

Data mining is to find hidden, effective, valuable, and understandable patterns from a large amount of unordered data, to find useful knowledge, to derive the trend and association of time, and to provide users with decision-making level decision-making support ability. The association rule mining algorithm based on the topology constraint performs hierarchical coding of each device in which each alarm occurs according to the hierarchical relationship between the network elements obtained by the established topology model. The connection relationship between the network elements reflected by the topology structure, combined with the propagation path of the fault, obtains the constraint condition of the association rule mining process. In the process of mining association rules, whether two or more items may be connected as a set of items is limited by such constraints. The interaction and mutual influence between network devices is the root cause of alarm propagation. Therefore, the patterns found in the alarm sequences sent by mutually influential devices are more targeted and more meaningful. If the relationship between devices is not introduced, the alarm of the related device cannot be filtered out, and a large number of meaningless modes are easily generated. Therefore, it is very important to introduce the constraints of network topology, and combining network topology constraints with data mining techniques can reduce the impact of noise and data loss by using constraints to find valuable rules [3].

Based on the summary and analysis of previous research results, this paper studies the network fault diagnosis of the embedded system method based on topology constraint and data mining. Firstly, by constructing a topology search algorithm, a fault diagnosis topology model is established, which eliminates the filtering of association rules without the relationship of topologies. Based on the collection of network alarm data, the quality of training samples is studied and related concepts are defined. The fault feature extraction algorithm is given, the hybrid system model is proposed, and the data mining model based on association rules is analyzed. The model algorithm is applied to the simulation experiment of network fault diagnosis of the embedded system. The algorithm in this paper provides a reference for further research on subsequent network fault diagnosis of the embedded system.

The article "Network Fault Diagnosis of Embedded System Based on Topology Constraint and Data Mining" was published in 2022. Journal: Comput Intell Neurosci.

## 2. Methods and Principles

### 2.1. Topology Constraint

The topology model is an abstract view of the network structure, which hides other aspects that are not related to the topology relationship. Through it, this relationship can intuitively understand the connection relationship of each network element in the network, discover the characteristics of the network connection, and study the network structure and network performance analysis and other aspects are very helpful.

The network topology model can filter out irrelevant alarm data through the topology relationship in the preprocessing stage. For a certain alarm to be analyzed in the original alarm data, the network element that uses the alarm finds all network elements or most network elements that have a topology relationship with the network element in the topology model and extracts the connected network elements. It is stored in a data structure and in the form of network elements to form a cluster of network elements. Under the framework of mean shift tracking, the target model and candidate target model are, respectively, written as follows [4]:

(1) $$\begin{array}{c} {\hat{q}}_{u}=C\sum_{i=1}^{n}k\left({\left\|x_{i}^{*}\right\|}^{2}\right)\delta \left[b\left(x_{i}^{*}\right)-u\right],\\ {\hat{p}}_{u}\left(y\right)=C_{h}\overset{n}{\underset{i=1}{\sum }}k\left({\left\|\frac{y-x_{i}}{h}\right\|}^{2}\right)\delta \left[b\left(x_{i}\right)-u\right], \end{array}$$

where *x*_*i*_^*∗*^ is the pixel in the target area, *x*_*i*_ is the pixel in the candidate target area with center *y*, *k* is the spatially weighted kernel function, and *b*(*x*_*i*_) is the histogram interval corresponding to the pixel at position *x*_*i*_.

The coefficient is used as a measure to measure the similarity between two eigenvectors of the target region and the candidate target region:

(2) $$\begin{array}{c} \hat{\rho }\left(y\right)=\overset{m}{\underset{u=1}{\sum }}\sqrt{{\hat{p}}_{u}\left(y\right){\hat{q}}_{u}}. \end{array}$$

The probability of crossover and mutation adopts an adaptive mechanism. As shown in (3) and (4), the probability of cross mutation is adjusted according to the individual fitness value so that poor individuals are more prone to cross mutation and good individuals are easy to save [5]:

(3) $$\begin{array}{c} P_{c}=\left\{\begin{array}{cc} P_{c2}-\frac{\left(P_{c2}-P_{c3}\right)\left(F{}^{\prime }-F_{\mathrm{avg}}\right)}{F_{\max}-F_{avg}}, & F{}^{\prime }\geq F_{\mathrm{avg}},\\ P_{c1}-\frac{\left(P_{c1}-P_{c2}\right)\left(F{}^{\prime }-F_{\min}\right)}{F_{\mathrm{avg}}-F_{\min}}, & F{}^{\prime }<F_{\mathrm{avg}}, \end{array}\right. \end{array}$$

(4) $$\begin{array}{c} P_{m}=\left\{\begin{array}{cc} P_{m2}-\frac{\left(P_{m2}-P_{m3}\right)\left(F-F_{\mathrm{avg}}\right)}{F_{\max}-F_{avg}}, & F{}^{\prime }\geq F_{\mathrm{avg}},\\ P_{m1}-\frac{\left(P_{m1}-P_{m2}\right)\left(F-F_{\min}\right)}{F_{\mathrm{avg}}-F_{\min}}, & F{}^{\prime }<F_{\mathrm{avg}}, \end{array}\right. \end{array}$$

where *F*_max_, *F*_min_, and *F*_avg_ are the maximum, minimum, and average fitness values of the population, respectively, *F*′ is the larger fitness value of the two individuals performing genetic manipulation, and there are *P*_*c*1_>*P*_*c*2_>*P*_*c*3_ and *P*_*m*1_>*P*_*m*2_>*P*_*m*3_.

The article "Network Fault Diagnosis of Embedded System Based on Topology Constraint and Data Mining" was published in 2022. Journal: Comput Intell Neurosci.

There is a certain model transformation relationship between the matching points in most images to be matched, and the topology relationship between several feature points in the same image is also approximately satisfied in the other image. For this purpose, the topology constraint can be performed by calculating the angle between the three feature points to purify the initial matching point. It is known that the coordinates of the three pairs of matching point pairs are (*x*_1_, *y*_1_)^*T*^, (*x*_2_, *y*_2_)^*T*^, (*x*_3_, *y*_3_)^*T*^ and (*x*_1_′, *y*_1_′)^*T*^, (*x*_2_′, *y*_2_′)^*T*^, (*x*_3_′, *y*_3_′)^*T*^, respectively, and the two angles *p* and *q* can be obtained by using the vector angle cosine formula [6]:

(5) $$\begin{array}{c} p=\arccos\left[\frac{\left(x_{1}-x_{2}\right)\cdot \left(x_{1}-x_{3}\right)+\left(y_{1}-y_{2}\right)\cdot \left(y_{1}-y_{3}\right)}{\sqrt{{\left(x_{1}-x_{2}\right)}^{2}+{\left(y_{1}-y_{2}\right)}^{2}}\cdot \sqrt{{\left(x_{1}-x_{3}\right)}^{2}+{\left(y_{1}-y_{3}\right)}^{2}}}\right],\\ q=\arccos\left[\frac{\left(x_{1}^{\prime }-x_{2}^{\prime }\right)\cdot \left(x_{1}^{\prime }-x_{3}^{\prime }\right)+\left(y_{1}^{\prime }-y_{2}\right)\cdot \left(y_{1}^{\prime }-y_{3}^{\prime }\right)}{\sqrt{{\left(x_{1}^{\prime }-x_{2}^{\prime }\right)}^{2}+{\left(y_{1}^{\prime }-y_{2}^{\prime }\right)}^{2}}\cdot \sqrt{{\left(x_{1}^{\prime }-x_{3}^{\prime }\right)}^{2}+{\left(y_{1}^{\prime }-y_{3}^{\prime }\right)}^{2}}}\right]. \end{array}$$

For the above algorithm, a set of relatively stable correct matching points need to be found as the initial point pair of the calculation. Therefore, the key step of the algorithm is to find a set of such points because only one group needs to be found in all the initial matching points. The point fits the requirements of calculation, so algorithm can search it by increasing the set conditions, and the specific implementation method will be shown in the following network topology model.

The article "Network Fault Diagnosis of Embedded System Based on Topology Constraint and Data Mining" was published in 2022. Journal: Comput Intell Neurosci.

### 2.2. Data Mining

Data mining technology is a database technology that extracts hidden, previously unknown, and potentially valuable knowledge and rules from vast amounts of data. The interest association rule directly indicates the recursive relationship between interests, and by simplifying the data in the buffer represented by the data model, it directly indicates the link relationship between the pages, which cannot directly reflect the degree of association between interests [7].

It is supposed that there are *n* learning samples, each with a set of observations (*x*_1_, *x*_2_,…, *x*_*m*_, *y*_*i*_^*∗*^) of *m*+1 parameters (*x*_1_, *x*_2_,…, *x*_*m*_, *y*_*i*_^*∗*^) · (*i*=1,2,…, *n*), *n* > *m*, and in practice, *n* is generally much larger than *m*, so as to ensure the accuracy and representativeness of the prediction results. The *n* learning samples of *m* parameters are defined as *n* vectors, that is, the expression of the learning sample is [8]

(6) $$\begin{array}{c} x_{i}=\left(x_{i1},x_{i2},\ldots ,x_{im},y_{i}^{*},\right),\;\left(i=1,2,\ldots ,n\right). \end{array}$$

Let *x*_0_ be the general form of a vector in (*x*_*i*1_, *x*_*i*2_,…, *x*_*im*_). The principle of the algorithms is the same, that is, to create an expression *y* = *y*(*x*_0_) and minimize its value:

(7) $$\begin{array}{c} \min\left(y\right)=\sum_{i=1}^{n}{\left[y\left(x_{0}\right)-y_{i}^{*}\right]}^{2}. \end{array}$$

In addition, algorithms are to establish an equation *y* = *y*(*x*_0_) to maximize the classification interval based on support vector points to get the optimal separation line. The accuracy of the results obtained is different because of the different methods used by these algorithms.

The data are preprocessed by the analytic hierarchy process to obtain the weights *W* of different nodes, and the order *S* of each node is obtained. The lower side correlation function is set as [9]

(8) $$\begin{array}{c} h_{mn}\left(z\right)=\left\{\begin{array}{cc} 0, & z\notin \left[z_{n}\left(1\right),z_{n}\left(2\right)\right],\\ \frac{z_{mn}-z_{n}\left(1\right)}{z_{n}\left(2\right)-z_{n}\left(1\right)}, & z\in \left[z_{n}\left(1\right),z_{n}\left(2\right)\right],\\ \frac{z_{n}\left(4\right)-z_{mn}}{z_{n}\left(4\right)-z_{n}\left(3\right)}, & z\in \left[z_{n}\left(3\right),z_{n}\left(4\right)\right], \end{array}\right. \end{array}$$

where *z*_*n*_(1) is the minimum value of the sample data, *z*_*n*_(2) = *z*_*n*_(3) is the number average, and *z*_*n*_(4) is the maximum number of data.

The article "Network Fault Diagnosis of Embedded System Based on Topology Constraint and Data Mining" was published in 2022. Journal: Comput Intell Neurosci.

The preprocessed sample data are *Z* = [*Z*(1) *Z*(2),...,*Z*(*M*)]*T*, and the information matrix H_*M*×*N*_ of (9) can be obtained via (8):

(9) $$\begin{array}{c} H_{M\times N}=\left[\begin{array}{cccc} h & h & \cdots & h\\ h & h & \cdots & h\\ \vdots & \vdots & \vdots & \vdots \\ h & h & \cdots & h \end{array}\right]. \end{array}$$

By *q*_*mn*_ = *h'*_*mn*_-*t*_*n*_+*ε* (*m* = 1, 2,...,*M* and *n* = 1, 2,...,*N*), *t*_n_ = min(h'_mn_), the negative number is shifted to a positive near zero number, the obtained positive matrix **Q**_*M*×*N*_^*n*^ is calculated as follows:

(10) $$\begin{array}{c} Q_{M\times N}^{n}=\left[\begin{array}{cccc} q_{11} & q_{12} & \cdots & q_{1N}\\ q_{21} & q_{22} & \cdots & q_{2N}\\ \vdots & \vdots & \vdots & \vdots \\ q_{M1} & q_{M2} & \cdots & q_{MN} \end{array}\right]. \end{array}$$

The association analysis method in data mining technology can be used for association discovery, sequence pattern discovery, and same time-series discovery. For the sake of simplicity, the transfer relationship between interest association rules cannot be considered when establishing interest association rules. For this simple interest association rule association model, using association discovery analysis method is more appropriate.

## 3. Topology Modeling Based on Fault Diagnosis

### 3.1. Topology Lookup Algorithm Implementation

At present, all network topology models have some shortcomings, especially the topology-level modeling research at the router level is still in its infancy, and the current research results and methods have yet to be enriched and developed. As seen above, as a typical representative of complex networks, the network topology has many basic parameters, such as node degree and its distribution, aggregation coefficient, median, and core number, but more importantly, new metrics to be discovered are metrics and network performance, such as synchronization performance and routing performance. The internal mechanisms of interaction between the two require further research by a large number of numerical simulations and empirical studies to provide a more in-depth qualitative and quantitative analysis of topology characteristics and metrics.

The network topology model lacks completeness for one or a few topology characteristics. In topology modeling, the existing research results show that model based on the design optimization principle is more consistent with topology structure than the scale-free model based on random principle. The network topology tree model used for topology lookup algorithm is shown in Figure 1. The network performance is also closer to the real network topology and the traditional scale-free model cannot be used to characterize the generation mechanism of network topology characteristics, such as robustness and vulnerability [10].

The article "Network Fault Diagnosis of Embedded System Based on Topology Constraint and Data Mining" was published in 2022. Journal: Comput Intell Neurosci.

In a complex or untreated network environment, due to network attacks, hardware errors, and environmental obstacles, data are prone to distortion or error during transmission or positioning [11]. This is different from simple errors that are easy to occur in ordinary networks, and the data will seriously affect the positioning result. The algorithm is characterized by maximizing the correlation between the signal space and the physical space after the data transformation and still retains the local spatial topology information. Therefore, the points adjacent to the coordinates are in the transformed signal space, and this paper focuses on the research of positioning methods in this network environment. This kind of erroneous data with serious deviations can also be called the wild value, and its value is greatly deviated from the collected normal data. In other words, this outlier feature makes the erroneous data far away from other normal data points in the geometric spatial distribution, thus having a lower distribution density, so the motivation for topology modeling is in the same dataset. The lower the point, the lower the impact on positioning to achieve better robustness.  Figure 2 is the topology analysis algorithm model flow.

The center position of the central core tracker is the initially selected center of the target area to be tracked; the target area of the start frame is manually given, the target area of the nonstart frame is obtained by tracking the previous frame image, and the border core tracker is the center position and is obtained by corner detection [4]. The corner point is a point where the gray level changes sharply in the image, and there are usually a large number of corner points at the boundary between the target and the background. The kernel tracking algorithm often uses the gray histogram to construct the target model, but the gray histogram is susceptible to image noise or changes, while the gradient direction histogram has the characteristics of being insensitive to the changes, which can be more robust. Target description is discussed, especially when the structure and gradient information of the tracking target is rich. Using these nuclear trackers at the target and background, the constructed kernel histogram contains both the target information and the relatively stable background information, which can improve the validity of the target model.

The article "Network Fault Diagnosis of Embedded System Based on Topology Constraint and Data Mining" was published in 2022. Journal: Comput Intell Neurosci.

### 3.2. Fault Diagnosis Topology Model

Fault diagnosis pattern recognition is an indispensable part of topology network fault diagnosis of the embedded system; the topology network can simulate the organization framework and construct a cognitive process to realize the fault handling. The working principle of this diagnostic method is to transmit the fault symptom to the system through the topology network and use the recognition model to classify the fault and obtain the diagnosis result. This type of diagnosis mainly uses the method of integrating the fault diagnosis data and, at the same time, training and practicing it. The data distributed in the topology network are expressed by means of computational translation, and finally, the fault diagnosis result is output. There are totally three algorithms which were compared in study, and they are diagnosis fault analysis system testing (DFAST), basic analysis system testing (BAST), and step fault analysis system testing (SFAST), respectively.

Topology networks can also integrate and collect ambiguous fuzzy fault information and integrate them into a complete fuzzy relational framework by means of mathematical logic such as functions. Different fault diagnosis topology model algorithm has different correct rates of retrieval under different window sizes, which has a significant impact on topology modeling (Figure 3). This framework can make unclear factors and avatars reasonable. In the scope, it provides a basis for network fault diagnosis of the embedded system. The diagnosis principle is mainly based on the integration of faults and the manifestation of form information, constructing a framework system belonging to the function, then focusing the fault factors and manifestations into a unified function framework, and using fuzzy relationship to carry out the fault factor category.

Network failures and signs of performance have strong uncertainties. The fuzzy relationship between the two makes it difficult to determine the cause of the two through common mathematical models, and the fuzzy logic network fault diagnosis of the embedded system method can be uncertain. The fault information is collected and integrated, and a relatively complete mathematical matrix model can be established through mathematical functions such as different functions. The establishment of the mathematical model can control the uncertain fault, and the symptom performance in a specific range and fault diagnosis provides a specific reference. The relationship between the cause and the symptom of the network system failure is extremely complicated and has strong randomness. Therefore, it is difficult to specifically locate the fault and analyze the cause by simply relying on the expert system. This kind of network diagnosis method can accurately judge the cause of the network failure and can bring some inspiration to the fault diagnosis of the maintenance personnel, but this method must be based on the establishment of a large fuzzy relational database and its intelligent learning ability.

The article "Network Fault Diagnosis of Embedded System Based on Topology Constraint and Data Mining" was published in 2022. Journal: Comput Intell Neurosci.

The optimization of the network topology determines the weight of the network, thus transforming the problem of the neural network into a hierarchical decentralized optimization problem with the layer of neurons. The correction of the decision-making scheme is through neural network learning and rough set learning. The exchange between the two is improved until the rough set learning selects the decision rule with the least attribute composition to correctly divide all the training set samples. Although the training sample set is the knowledge given by the domain experts, including the knowledge formed by the fault condition attribute, there are inevitably incompatible situations, which will produce redundant samples. Training such samples will not only improve the correctness of decision-making but also reduce the learning efficiency of neural networks. On the contrary, each attribute of the fault symptom subset has different contributions to decision-making. The system needs to reflect the importance of different attributes in the learning process to improve learning efficiency [12].

## 4. Analysis of Alarm Data Based on Data Mining

### 4.1. Network Alarm Data Collection

Data extraction is the primary task of data analysis and the extracted data mainly includes alarm standardization data and network management system alarm data. It should be noted that the specific time zone should be specified before extracting data, and then, the time zone is determined by the network management system, and all alarm data in the data are extracted. After excluding the interference of the special data, the valuable data need to be filtered from the remaining data, and the interference alarm is removed. At the same time, the standardization field of the alarm information is set to the classification class and the weight class to judge the value of the alarm information. In order to avoid this problem, the predecessor proposed that, in the fault feedback phase, a mobile sensor node is set in the detection area, and the mobile sensor node starts from the base station, collects the state information of all the sensor nodes by the mobile, and transmits to the base station. Finally, the selected valuable alarm information is integrated to form a network alarm data center.

The article "Network Fault Diagnosis of Embedded System Based on Topology Constraint and Data Mining" was published in 2022. Journal: Comput Intell Neurosci.

If each node communicates with the base station, the node farther from the base station needs to communicate with the base station by means of the multihop node, which increases the energy consumption of the sensor node and is prone to error during transmission [13]. After obtaining all the data in the specified time period, the data should be cleaned, and the abnormal data, the missing data, the erroneous data, and the duplicate data, which affect the accuracy of the analysis, are eliminated, thereby ensuring the quality of the data analysis and realizing the accurate analysis of alarm information (Figure 4). Since the wireless sensor node has a certain communication range, it is not necessary to traverse each sensor node when performing fault feedback. The area where the sensor node is located can be divided and then the mobile sensor node can traverse each small area.

In the alarm association, the association analysis of the alarms can be used to obtain the strong association alarm rules with different support degrees and confidence levels. The minimum support degree and the minimum confidence level are used to help mine the root cause alarms to determine the alarms in the frequent alarm transaction set. In addition, we only specify the weight of the minimum support, the frequent item sets are filtered out, and all the confidences of the alarm associations under the frequent item sets are retained [14]. The purpose of this is mainly as follows: on the one hand, the frequent item sets in the massive alarm data can be filtered out as the target transaction set for determining the alarm weight by specifying the minimum support; on the other hand, all the alarm associations are retained. The confidence level can compare the relationship between all alarms' events in an alarm transaction set to determine the weight of each alarm event.

The core idea of the police weighting process of the big number theorem is to frequency the alarm weights, that is, according to the confidence level and alarm level of the alarm association rules, the alarm transaction set is taken as a set, and each alarm event is used as a random event through a large-scale simulation which calculates the frequency value of each alarm event occurring in this set as a weight. Alarm correlation analysis is a key issue in fault management, which helps network administrators delete a large number of redundant alarms, analyze the cause of the fault, and predict the occurrence of the fault. The traditional correlation analysis method mainly acquires relevant knowledge through experts, so it cannot meet the needs of network maintenance under the characteristics of large-scale, complex, and heterogeneous network, and the data mining method can make up for this deficiency.

The article "Network Fault Diagnosis of Embedded System Based on Topology Constraint and Data Mining" was published in 2022. Journal: Comput Intell Neurosci.

### 4.2. Association Rule Mining Model

The association rules are different from the traditional association rules. The reliability of each item included in the requirements of the trusted association rules is in the same order of magnitude and does not care about the size of the entire rule. The redefinition of confidence can reflect the credibility of the rules, and traditional support can no longer be considered. For the mining of trusted association rules, the algorithm uses the adjacency matrix to generate two trusted sets and then uses the maximal group idea to generate all trusted association rules, thus avoiding scanning the database multiple times. These new metrics are designed to reduce the generation of false rules. Combining them into the generation process of frequent item sets can greatly compress the number of candidate sets generated and can mine strong intimacy association patterns. However, most of these methods are still based on algorithms, not only to scan the database multiple times but also to discriminate the interest of each candidate, so the time performance is low.

When constructing the sample set, a certain number of records before and after each fault occurrence time point are used as fault samples, and the nonfault time records are divided into several normal samples, and the normal sample records are the same as the fault samples. Firstly, the dataset is preprocessed, and the feature and constructor vector are extracted; then, the network model is built, the model parameters are configured, and the network training is performed. After the requirements are met, the network parameters are saved and the trained model is output. When there is new sample data to be diagnosed, the data are input into the trained network model, and the fault diagnosis result is fault or normal.

Depending on whether duplicates of the same dimension are allowed, multidimensional association rules can be subdivided into interdimensional association rules and hybrid dimension association rules, allowing dimensions to appear simultaneously on the left and right sides of the rules. Relationship between node and node degree, node failure rate, and diagnostic accuracy are shown in Figure 5. Dimensional association rules and mining of multidimensional association rules also need to consider different types of fields, namely, category data and numerical data. For category data, the general association rule algorithm can handle it, while the logarithmic data need to be converted into category data for processing. Numeric fields are divided into predefined hierarchies; these intervals are all predefined by the user, and the resulting rule is also called the static quantity association rule [15, 16].

The article "Network Fault Diagnosis of Embedded System Based on Topology Constraint and Data Mining" was published in 2022. Journal: Comput Intell Neurosci.

The algorithm is the most influential algorithm for mining a completely frequent item set and the algorithm has two key steps: one is to find all frequent item sets and the other is to generate strong association rules [17–19]. The algorithm is also a breadth-first algorithm, and the algorithm is based on the a priori algorithm. The first method of the algorithm uses the a priori algorithm when scanning the database. When scanning again, it is no longer scanning the entire database, but only scanning the candidate set generated last time. The scanning also calculates the support of frequent item sets to reduce the support, and the time to scan the database is to improve the efficiency of the algorithm; the fusion of algorithm produces algorithm. When the database is initially scanned, a priori algorithm is used. When the generated candidate set size can be stored in memory for processing, it will be transferred to algorithm until all frequent item sets are found.

The entire process only needs to scan the database twice, but the number of candidate sets generated is relatively large and the algorithm also adopts the idea of database partitioning. The database is divided into several partitions and marked at the beginning of each partition. In the process of scanning the database, a candidate set can be added to the marked points of each partition, and parallel calculation is performed when calculating the item set. Discovering frequent item sets is a key step in mining association rules. The algorithm also utilizes that the subset of frequent item sets is a frequent item set, and the super set of infrequent item sets is a nonfrequent item set, and this property effectively prunes frequent item sets.

## 5. Algorithm Simulation and Analysis

Since there is no link in the algorithm logic that combines the frequent patterns of item generation by the frequent patterns of the items in the classical algorithm, the tree structure is used for mining, that is, after the tree is generated, the frequent pattern can be generated in one step. Therefore, the network topology constraint is added after the algorithm generates all the frequent patterns, that is, after the algorithm digs out the frequent patterns, they are sequentially determined whether the network topology constraints are met, and then, the nonconforming patterns are deleted from the final frequent pattern set. Such an operation can avoid the infrequently frequent patterns being delivered to the user as the final output, which is more beneficial to the actual needs of the user.

The article "Network Fault Diagnosis of Embedded System Based on Topology Constraint and Data Mining" was published in 2022. Journal: Comput Intell Neurosci.

The experimental results show that the network fault diagnosis of the embedded system method based on convolutional neural network can achieve better results than the traditional naive logistic regression and multilayer perception methods in the same training set and test set. Compared with the traditional network fault diagnosis of the embedded system method, the method based on convolutional neural network is simpler, no need to artificially extract the features in the text, and the network model configuration is simple, and the training data amount and model training time are reduced, and the matching calculation is reduced.

The topology search algorithm mainly constructs the classifier by discovering the association rules in the training set. Relationship between the remaining alarm number and the matching threshold value under different sliding steps is different from each other (Figure 6). In the construction process of the decision tree, the most time-consuming operation is to perform statistical calculation of the class distribution information on the dataset belonging to each nonterminal node and to split the dataset by using the splitting criterion. The discovery of association rules uses a classical algorithm that is effective for discovering association rules that are hidden among a large number of transaction records. However, when using it to discover classification rules, in order to prevent some rules from being missed, the minimum support is often set to zero. At this time, the algorithm cannot play its optimization role. As a result, the frequent sets generated sometimes cannot be in memory accommodated so that the program cannot continue to run. The method uses a group-based counting method to collect the category distribution information of various attribute value combinations in the training set and finds meaningful classification rules through the two thresholds of minimum confidence and minimum support.

In order to diagnose and analyze network faults based on data mining, it is necessary to first obtain information that reflects the relevant state of the network to a certain extent. Only the more completed and comprehensive the information of the relevant network state can be related. In actual network management, information exchanges between different management domains are relatively small due to security and other factors. The fault information is more included, which is more conducive to the discovery and resolution of faults. If designers want to fully obtain relevant network information, they need to refer to the network management of the computer and related diagnostic tools for network failure and refer to how it provides relevant data. The statistical content in the network device can be obtained by performing certain accesses to related data items. After that, comprehensive analysis of the statistical contents of multiple related network devices can be carried out to realize the basic management of the network.

The article "Network Fault Diagnosis of Embedded System Based on Topology Constraint and Data Mining" was published in 2022. Journal: Comput Intell Neurosci.

From the perspective of data mining, data warehouse is the platform for data mining implementation and data mining is an analysis and the decision-making method. Based on the principles of artificial intelligence, machine learning, and statistics, it analyzes and mines historical data based on data warehouses or data marts to find out the relationship patterns hidden in these data. It reflects the intrinsic nature of the data and makes a higher level of abstraction of the information contained in the data. The data mining process is divided into the following stages: data preparation, data selection, preprocessing, data reduction, target determination, algorithm determination, data mining, and pattern recognition and knowledge evaluation. The first four stages complete the data warehouse to prepare for knowledge discovery and five stages to mine useful knowledge. Data warehousing and data mining are inextricably linked and a typical data warehouse mainly includes data import, data warehouse and data mart, and access tools. The application of data warehouse and data mining technology in the field of remote monitoring and fault diagnosis greatly improves the efficiency and depth of data analysis and provides a powerful means for intelligent fault diagnosis, especially fault prediction, so that remote equipment enjoys the expert level.

According to the mining technology, the associated rules reflect certain dependencies or some related knowledge between certain things. If there are two or more related relationships, any one of them can be certain predictions based on other attributes and use the four related parameters of confidence, support, minimum confidence, and minimum support to determine the next rule so that obstacle data that are not yet known according to this rule can be determined. Relationship between the remaining warning number and regular association number under different algorithms is shown in Figure 7. This standard also stipulates the items and types of data that must be used for the agent of the network, as well as the agents that allow the operation of the network. The extraction is performed and quantified accordingly to form a global network alarm model.

The article "Network Fault Diagnosis of Embedded System Based on Topology Constraint and Data Mining" was published in 2022. Journal: Comput Intell Neurosci.

Centralized fault diagnosis is not a good solution, and data mining cannot be performed based on alarm information in real time. Researching distributed real-time fault diagnosis algorithms is of great theoretical value and practical significance for better reducing the time of system faults and improving the accuracy of fault location. Because different network equipment vendors do not agree on the alarm format and content and combine the characteristics of related network alarms, this paper first deals with the network alarm information, according to the characteristics of network alarms and related rules to carry out key attributes.

## 6. Conclusions

This paper studied the network fault diagnosis of the embedded system method based on topology constraint and data mining. Firstly, a fault diagnosis topology model was established by constructing a topology search algorithm, which eliminated the filtering of association rules without topology relationship; the association rule-based data mining model was analyzed through the collection of network alarm data; the model algorithm was applied to the simulation experiment of network fault diagnosis of the embedded system and achieved good results. A new neural network algorithm based on rough set decision is proposed and the corresponding network fault is designed. A diagnostic model that manages all subnets and managed devices by providing a single network operation control environment is in a mixed network environment. The causes of noise data are data false alarms and measurement errors. When the fault occurs, the data of some variables of the system will fluctuate greatly, and some properties of the constructed network model will also change. The results show that correcting rage of retrieval varies from 0.65 to 090 under different window size; the running time of the proposed method drops from 310 s to 35 s during 1–8 step/s of the sliding step, while the node degree ranges from 8 to 14 and diagnostic accuracy ranges from 0.97 to 0.94; the remaining alarm number increases from 0.5 to 3.5 threshold value, while the regular association number is distributed in an interval of 40 to 140. The algorithm in this paper provides a reference for further research on network fault diagnosis of the embedded system. Moreover, further research studies should focus on the detailed influence of embedded system's inner structures on network fault diagnosis based on topology constraint and data mining.

## Figures and Tables

**Figure 1:** Network topology tree model used for topology lookup algorithm.

**Figure 2:** Topology analysis algorithm model flow.

**Figure 3:** Correct rate of retrieval under different window sizes.

The article "Network Fault Diagnosis of Embedded System Based on Topology Constraint and Data Mining" was published in 2022. Journal: Comput Intell Neurosci.

**Figure 4:** Relationship between algorithm running times and sliding step (a) and alarm number (b).

**Figure 5:** (a) Relationship between node and node degree. (b) Node failure rate and diagnostic accuracy.

**Figure 6:** Relationship between the remaining alarm number and the matching threshold value under different sliding steps.

**Figure 7:** Relationship between the remaining warning number and regular association number under different algorithms.

## Data Availability

The data used to support the findings of this study are available from the corresponding author upon request.
